RETRACTED

# Experimental Infection of Mice with Avian Paramyxovirus Serotypes 1 to 9

**DOI:** 10.1371/journal.pone.0016776

**Published:** 2011-02-10

**Authors:** Sunil K. Khattar, Sachin Kumar, Sa Xiao, Peter L. Collins, Siba K. Samal

**Affiliations:** 1 Virginia-Maryland Regional College of Veterinary Medicine, University of Maryland, College Park, Maryland, United States of America; 2 Laboratory of Infectious Diseases, National Institute of Allergy and Infectious Diseases, National Institutes of Health, U.S. Department of Health and Human Services, Bethesda, Maryland, United States of America; University of Kansas Medical Center, United States of America

## Abstract

The nine serotypes of avian paramyxoviruses (APMVs) are frequently isolated from domestic and wild birds worldwide. APMV-1, also called Newcastle disease virus, was shown to be attenuated in non-avian species and is being developed as a potential vector for human vaccines. In the present study, we extended this evaluation to the other eight serotypes by evaluating infection in BALB/c mice. Mice were inoculated intranasally with a prototype strain of each of the nine serotypes and monitored for clinical disease, gross pathology, histopathology, virus replication and viral antigen distribution, and seroconversion. On the basis of multiple criteria, each of the APMV serotypes except serotype 5 was found to replicate in mice. Five of the serotypes produced clinical disease and significant weight loss in the following order of severity: 1, 2>6, 9>7. However, disease was short-lived. The other serotypes produced no evident clinical disease. Replication of all of the APMVs except APMV-5 in the nasal turbinates and lungs was confirmed by the recovery of infectious virus and by substantial expression of viral antigen in the epithelial lining detected by immunohistochemistry. Trace levels of infectious APMV-4 and -9 were detected in the brain of some animals; otherwise, no virus was detected in the brain, small intestine, kidney, or spleen. Histologically, infection with the APMVs resulted in lung lesions consistent with broncho-interstitial pneumonia of varying severity that were completely resolved at 14 days post infection. All of the mice infected with the APMVs except APMV-5 produced serotype-specific HI serum antibodies, confirming a lack of replication of APMV-5. Taken together, these results demonstrate that all APMV serotypes except APMV-5 are capable of replicating in mice with minimal disease and pathology.

## Introduction

The family *Paramyxoviridae* is large and diverse and includes viruses that have been isolated from a wide variety of mammalian and avian species around the world [1]. Some members of the family are responsible for major human and animal diseases, while others cause inapparent infections. The viruses belonging to this family are pleomorphic and enveloped and contain a non-segmented, negative-sense, single-stranded RNA genome of 13–19 kb. On the basis of virus structure, genome organization and sequence relatedness, the family *Paramyxoviridae* is divided in to two subfamilies: *Paramyxovirinae and Pneumovirinae* [1]. The subfamily *Paramyxovirinae* is divided into five genera: *Respirovirus* (including Sendai virus and human parainfluenza virus types 1 and 3), *Rubulavirus* (including simian virus type 5, mumps virus, and human parainfluenza virus types 2 and 4), *Morbillivirus* (including measles and canine distemper viruses), *Henipavirus* (comprising Hendra and Nipah viruses), and *Avulavirus* (comprising the avian paramyxoviruses [APMVs]). Subfamily *Pneumovirinae* contains two genera, *Pneumovirus* (including human respiratory syncytial virus and bovine respiratory syncytial virus) and *Metapneumovirus* (comprising human metapneumovirus and the avian metapneumoviruses) [1], [2].

RETRACTED

All the paramyxoviruses isolated from avian species are classified into genus *Avulavirus*, representing the APMVs, and genus *Metapneumovirus*, representing the avian metapneumoviruses. The APMVs have been divided into nine serotypes (APMV 1 to 9) based on hemagglutination inhibition (HI) and neuraminidase inhibition (NI) assays [3]. Recently, APMVs were isolated from Rockhopper Penguins in the Falkland Islands. Serological and genome characterizations suggested that these viruses probably represent a new serotype (APMV-10) [4]. APMV-1, which includes all strains of NDV, has been extensively characterized because virulent NDV strains are important causes of disease in chickens. Complete genome sequences have been determined for a number of NDV strains, and there is extensive information on NDV molecular biology and pathogenesis [5]–[15]. Comparatively little is known about the other eight APMV serotypes. As an initial step towards their characterization, complete genome sequences of APMV serotypes 2 to 9 were recently determined [16]–[26].

APMV-1 (NDV) strains are divided into three pathotypes: highly virulent (velogenic) strains that cause severe respiratory and neurologic diseases in chickens; moderately virulent (mesogenic) strains that cause milder disease, and nonpathogenic (lentogenic) strains that cause inapparent infection. In contrast, much less is known about the biological characteristics and pathogenicity of APMV-2 to -9. APMV-2 has been associated with severe respiratory disease and drop in egg production in turkeys [27], [28]. APMV-3 has been associated with encephalitis and high mortality in caged birds, respiratory diseases in turkeys and stunted growth in young chickens [29], [30]. APMV-5 causes disease in budgerigars that is characterized by depression, dyspnoea, diarrhea and high mortality [31]. APMV-6 and -7 cause mild respiratory disease in turkeys and are associated with a drop in egg production [32]–[34]. APMV-4, -8, and -9, isolated from ducks, waterfowl, and other wild birds did not produce any clinical signs of viral infection in chickens [35]–[39]. Recently, we performed experimental infection of 1-day-old chicks and 4-week-old chickens and turkeys with APMV-2 strains, Yucaipa and Bangor, and documented viral infection in the gastrointestinal and respiratory tracts [40]. We also performed experimental infection of 2-week-old chickens and turkeys with APMV-3 strains, Netherlands and Wisconsin, and documented viral infection in the brain, lungs, spleens, trachea, pancreas and kidney [41].

RETRACTED

In the last 10 years, reverse genetic techniques have made it possible to engineer NDV as a potential vaccine vector for delivery of a number of foreign antigens not only in avian hosts but also in murine and nonhuman primate models [42]–[50]. In addition, NDV has been evaluated as a promising broad spectrum oncolytic agent in a mouse model [51]–[54]. Safety of different strains of NDV, due to attenuation by host range restriction, has been documented in these animal models [55]. In the future, we plan to use reverse genetic techniques to evaluate other APMV serotypes (serotype 2 to 9) as vaccine vectors and oncolytic agents. However, small laboratory animal models will be needed to evaluate their replication, immunogenicity and safety. In the current study, we sought to evaluate mice as a small animal model for infection with APMV 2 to 9. We inoculated BALB/c mice intranasally with APMV serotypes 1 to 9 and monitored clinical signs and viral replication and tropism in a number of possible target organs. We further studied the serological responses to APMV infection in these animals. The results showed that BALB/c mice are susceptible to infection with all of the APMV serotypes except serotype 5. Viral replication occurred mostly in the upper and lower respiratory tracts. The data generated using this animal model will be helpful in elucidating mechanisms of immunity and pathogenesis and evaluating candidate recombinant vaccines.

## Materials and Methods

### Cells and viruses

Chicken embryo fibroblast (DF1) and African green monkey kidney (Vero) cell lines, obtained from the American Type Culture Collection (ATCC, Manassas, VA), were grown in Dulbecco's modified Eagle medium (DMEM) containing 10% fetal bovine serum (FBS) and maintained in DMEM with 5% FBS. The prototype strains of all nine APMV serotypes used in this study were: APMV-1 strain LaSota/46, APMV-2 strain chicken/Yucaipa/California/56, APMV-3 strain parakeet/Netherland/449/75, APMV-4 strain duck/Hongkong/D3/75, APMV-5 strain budgerigar/Kunitachi/74, APMV-6 strain duck/HongKong/18/199/77, APMV-7 strain dove/Tennessee/4/75, APMV-8 strain goose/Delaware/1053/76, and APMV-9 strain duck/New York/22/78. All of the strains except for serotype 5 were obtained from National Veterinary Services Laboratory, Ames, Iowa. APMV-5 strain budgerigar/Kunitachi/74 was kindly provided by Dr. Ian Brown, the Veterinary Laboratories Agency, Weybridge, Surrey, UK. All of the APMV serotypes except serotype 5 were grown in the allantoic cavity of 9-day-old specific-pathogen-free (SPF) embryonated chicken eggs. APMV serotype 5 was grown in Vero cells. The allantoic fluids from infected eggs were collected 96 h post-inoculation and virus titers were determined by hemagglutination (HA) assay with 0.5% chicken RBC. In the case of APMV-5, the titer was determined by plaque assay on Vero cells. The APMV-5 samples were inoculated in triplicate onto 24-well plates of Vero cells at 80% confluency, incubated for 1 h, washed with PBS, overlaid with 0.8% methylcellulose, and observed for plaque production until 7 days post inoculation (dpi). The cells were fixed with methanol and stained with 1% crystal violet. Values for each tissue sample were based on average plaque count from three wells.

RETRACTED

### Preparation of hyperimmune antiserum against the viral nucleocapsid (N) protein of each serotype of APMV

Each APMV serotype strain described above was purified on a sucrose gradient and the virion proteins were separated on a 10% SDS-polyacrylamide gel and negatively stained using E-Zinc TM reversible stain kit (Pierce, Rockford, IL). The N protein specific band was excised from the gel and destained with Tris-glycine buffer pH 8. The excised gel band was minced in a clean pestle and mixed with elution buffer (50 mM Tris-HCl buffer pH 8, 150 mM NaCl, 0.5 mM EDTA, 5 mM DTT and 0.1% SDS) and transferred to the upper chamber of a Nanosep centrifugal device (Pall Life Sciences, Ann Arbor, MI, USA). After centrifugation two times, the eluted protein in the supernatant was quantified and 0.2 mg of protein was mixed with complete Freund's adjuvant and injected subcutaneously into a rabbit. After two weeks, a booster immunization was given with 0.2 mg of protein mixed with incomplete Freund's adjuvant and 2 weeks later the hyperimmune sera were collected. The sera were tested by Western blot and were found to recognize specifically the N protein of the respective APMV serotypes (data not shown).

RETRACTED

### Experimental infection of Mice

BALB/c mice aged 4 weeks, of either gender, were obtained from Charles River Laboratories, Wilmington, Massachusetts. Mice were housed in microisolator cages in our Bio Safety Level-2 facility and provided water and food ad libitum. Mice were housed in groups of 6 for inoculation of each APMV serotype. Mice were anaesthetized by isofluorane and inoculated intranasally with 50 µl of freshly harvested allantoic fluid containing 2^7^ HA units of each APMV serotype, except for serotype 5 which contained 3×10^3^ PFU/ml of cell culture harvested virus. A group of 6 mice was mock infected with normal allantoic fluid. Mice were weighed and examined two times daily for clinical signs, change in activity and behavior. Three mice from each group were euthanized at 3 day post inoculation (dpi) and other three at 14 dpi by CO_2_ asphyxiation. Necropsies were performed immediately and tissues from lung, nasal turbinate, brain, small intestine, kidney and spleen were collected. One half of each tissue sample was immediately processed for virus detection and quantification and the other half was stored in 10% neutral buffered formalin for histopathology and immunohistochemistry experiments. On 14 dpi, blood was collected from each mouse just before euthanasia and sera were prepared for analysis. All the animal research was conducted according to the guidelines approved by Institutional Animal Care and Use Committee of the University of Maryland. The protocol number is R-09-47 [Immunogenicity and protection efficacy of recombinant NDV expressing foreign antigens in mammalian models (mice and ferrets)].

### Virus detection and quantification

Tissues collected from different organs were homogenized in 1 ml of ice-cold DMEM. Tissue homogenates were centrifuged at 4°C for 10 min at 1000× g and supernatants were collected. For virus detection, 100 µl of clarified homogenate from each tissue was injected into allantoic cavities of five 9-day-old embryonated SPF chicken eggs. Eggs were incubated at 37°C for 4 days. Allantoic fluid was collected from each egg and the presence of virus was detected by hemagglutination (HA) test. For quantification of virus, clarified homogenate from each tissue was diluted in serial 10-fold dilutions in DMEM. The dilutions were inoculated in triplicate onto DF1 cell monolayers in 96-well plates and incubated at 37°C for 1 h. The wells were overlaid with 0.8% methylcellulose in DMEM supplemented with 10% normal allantoic fluid and 2% FBS and incubated at 37°C in a CO_2_ incubator for 4 days. The monolayers were washed with PBS, permeabilized with 100% cold methanol, and incubated with a 1∶300 dilution of primary N-specific antibody in PBS produced as described above. After three washes with PBS, plates were incubated with a 1∶1000 dilution of secondary antibody (Alexa Fluor 488 conjugated goat anti rabbit immunoglobulin G antibodies). After a further wash cycle, plates were viewed under a fluorescent microscope and fluorescent foci were counted.

RETRACTED

### Histopathology and Immunohistochemistry

Tissues from infected and control mice were examined by histopathology and immunohistochemistry. Paraffin embedded sections of all the tissues were prepared at Histoserve, Inc. (Maryland, USA). The 5 micron tissue sections were stained with hematoxylin and eosin for histopathology. The severity of inflammation in lungs and nasal turbinate of each APMV infected mouse was assessed based on the extent of fibrin, edema, and mixed inflammatory cells (neutrophils, macrophages, lymphocytes, plasma cells), necrotic cellular debris, and hemorrhage in alveolar spaces and septae.

Immunohistochemical staining was performed on lung and nasal turbinate tissues to detect viral N protein using the following protocol. Briefly, tissue sections were deparaffinized in 2 changes of xylene (5 mins each) and hydrated by incubation in 2 changes each of 100% (3 mins each), 95% (1 min each), and 80% (1 min each) ethanol followed by washing in distilled water. Slides were heated for 40 mins in a staining dish containing sodium citrate buffer (10 mM citric acid, 0.05% Tween 20, pH 6.0) until the temperature reached 95–100°C, followed by cooling to room temperature. Sections were washed two times in PBS-Tween 20 for 2 min each, blocked with 2% normal goat serum in PBS for 30 mins, and incubated with 1∶200 dilution of primary antibody (hyperimmune sera raised against N protein of a particular APMV serotype) in PBS for 1 h at room temperature. The sections were washed three times with PBS-Tween 20 for 2 min each and incubated with 1∶1000 dilution of secondary antibody (Alexa Fluor 488 conjugated goat anti rabbit immunoglobulin G antibodies) in PBS for 1 h. After a further wash cycle, the sections were mounted with glycerol and viewed under fluorescent microscope.

### Serological analysis

The antibody levels in serum samples collected from mice infected with APMVs on 14 dpi, were evaluated by hemagglutination inhibition (HI) assay except in the case of APMV-5 [56]. In our standard HI assay, the normal mice sera produced nonspecific HI. Therefore a modified HI assay was used. Briefly, 25 µl of mice serum was first treated with 50 µl of receptor destroying enzyme II (catalog number YCC 340–122; Accurate Chemical and Scientific, Westbury NY) at a 1∶3 ratio (vol/vol) at 37°C overnight. Then 25 µl of 5% sodium citrate was added and incubation was continued at 56°C for 30 min. Each serum sample was allowed to cool to room temperature and 100 µl of packed chicken RBCs were added. After incubation at 4°C for 30 min, samples were centrifuged at 1000× g for 10 min. Supernatants were used for HI assay. For the HI assay, twofold serial dilutions of treated sera (50 µl) were prepared, and each dilution was combined with 4 HA units of a particular APMV serotype. Following 1 h of incubation, 50 µl of 1% chicken RBC was added and incubated for 30 min at room temperature, and hemagglutination was scored. In the case of APMV-5, antibody titers were measured by a plaque reduction assay. Briefly, the sera were heat inactivated at 56°C for 30 mins. Ten-fold dilutions of sera were made and mixed with a constant amount of APMV-5 (3×10^3^ PFU), and incubated at room temperature for 1 h in a shaker. The antigen antibody mixtures were analyzed by plaque assay as described above. The serum titer that reduced plaque numbers by 70% was the end point titer.

RETRACTED

## Results

### Clinical disease and gross pathology

Four-week-old BALB/c mice in groups of six were inoculated by the intranasal route with 2^7^ HA units of APMV serotypes 1 to 9 except in the case of serotype 5, for which 3×10^3^ PFU/ml of virus were inoculated. Three animals from each group were sacrificed 3 dpi, and the remaining three were sacrificed 14 dpi. None of the mice infected with APMV serotypes 3, 4, 5 and 8 displayed any overt clinical signs and loss of weight (Fig. 1). At 1 dpi, the mice infected with APMV serotype 1 and 2 had a pronounced decrease in their physical activity, a tendency to huddle and very ruffled fur compared to control mice. The mice infected with APMV serotypes 6, 7 and 9 also presented these clinical signs, which were less marked than those of the mice infected with serotypes 1 and 2. Mice infected with serotypes 1 and 2 exhibited more weight loss than mice infected with serotypes 6, 7 and 9. The loss in weight was observed until day 4 in mice infected with serotypes 1 and 2, until day 3 in mice infected with serotypes 6 and 9, and until day 2 in mice infected with serotype 7. Further, the weight gain remained poor in mice infected with serotypes 1 and 2 after 4 dpi. None of the mice infected with serotypes 1 to 9 died of disease. When the animals were sacrificed 3 dpi and 14 dpi, the following tissues were collected: lung, nasal turbinate, brain, spleen, kidney and small intestine. In all cases, gross examination revealed normal tissue morphology with no noticeable gross lesions.

**Figure 1:** Weight loss in mice infected with APMV serotypes 1 to 9. Mice in groups of 6 were inoculated with allantoic fluid containing 2^7^ HA units of each APMV serotype except serotype 5, which contained 3×10^3^ PFU/ml of cell culture harvested virus. The control group was inoculated with normal allantoic fluid. The mice were weighed daily and weight lost was calculated as a percent of the weight on day 0. Data depict the mean ± SD from 3 mice per group.

RETRACTED

### Virus isolation and titration in tissue samples

To determine the sites of APMV replication, one half of each sample of lung, nasal turbinate, brain, spleen, kidney and small intestine tissue collected 3 dpi and 14 dpi was homogenized and clarified supernatants were prepared. For each of the serotypes except APMV-5 (which does not grow in the allantoic cavity of eggs), aliquots were inoculated into the allantoic cavity of embryonated 9-day-old chicken eggs, and 4 dpi the allantoic fluid was collected and assayed for virus infection by HA test (Table 1). For all of the serotypes of APMV except serotype 5, virus was detected from the lungs and nasal turbinates at 3 dpi. APMV serotypes 4 and 9 also were detected in the brain in two mice each at 3 dpi. Virus was not detected in any other tissues isolated 3 dpi, or in any tissue isolated 14 dpi.

**Table 1:** Virus isolation from the indicated tissue harvested from mice 3 dpi with APMV serotypes 1 to 9*.

APMV Serotype	Lung	Nasal turbinate	Spleen	Kidney	Small intestine	Brain
**1**	+++	+++	-	-	-	-
**2**	+++	+++	-	-	-	-
**3**	+++	+++	-	-	-	-
**4**	+++	+++	-	-	-	++
**5**	ND	ND	ND	ND	ND	ND
**6**	+++	+++	-	-	-	-
**7**	+++	+++	-	-	-	-
**8**	+++	+++	-	-	-	-
**9**	+++	+++	-	-	-	++

* Mice in groups of 3 were inoculated with 50 ìl of allantoic fluid containing 2^7^ HA units of each APMV serotype except serotype 5, which contained 3×10^3^ PFU/ml of cell culture harvested virus. The control group was inoculated with normal allantoic fluid. Tissues were harvested 3 dpi and homogenized, and clarified supernatant fluid was inoculated into 9-day-old embryonated eggs and tested for virus 4 days later by HA assay.

+  = each + indicates isolation of virus from one mice.

-  = no virus was isolated.

ND = not detected.

For quantification of the replication of each APMV, homogenates of tissue samples that were positive for virus isolation in eggs were used to generate 10-fold dilution series that were inoculated onto chicken DF1 cells and incubated under methylcellulose overlay. The tissue homogenates from APMV-5-infected mice were analyzed in parallel. Immunofluorescence staining for the N protein 4 dpi revealed foci with strong positive intracellular staining in the case of samples from the lungs and nasal turbinates for each of the APMV serotypes except APMV-5, for which no virus was detected (Fig. 2). The mean virus titers from lungs of the mice infected with APMV serotypes 1, 2, 3, 4, 6, 7, 8 and 9 were 2×10^2^, 3×10^2^, 7×10^1^, 2×10^2^, 2×10^2^, 3×10^1^, 5×10^2^ and 9×10^2^, respectively (Table 2). The mean virus titers from nasal turbinates of the mice infected with APMV serotypes 1, 2, 3, 4, 6, 7, 8 and 9 were 3×10^1^, 6×, 2×10^1^, 1×10^2^, 3×10^2^, 1×10^1^, 2×10^2^ and 8×10^2^, respectively. These results indicated the titer of APMV serotype 9 was higher than other serotypes in the lung and nasal turbinates, suggesting that it was the most permissive APMV for replication in mice. The brain tissue samples of APMV serotypes 4 and 9 infected mice that were positive for infection of embryonated eggs were negative in cell culture. No virus was detected in any sample from day 14, indicating viral clearance. The APMV-5 samples also were inoculated onto African green monkey Vero cells, where no virus could be detected from any of the tissue harvested from mice 3 dpi or 14 dpi by immunofluorescence staining. This indicated that APMV-5, alone among the APMV serotypes, was not recoverable from infected mice.

RETRACTED

**Figure 2:** Immunofluorescence visualization of foci formed in DF-1 cells infected with each of the 9 APMV serotypes. Mice were infected with each of the APMV serotypes and lungs were harvested 3 dpi and homogenized, and the clarified supernatants were inoculated onto DF-1 cells that were incubated 4 days under methycellulose prior to immunostaining with polyclonal antiserum specific to the N protein of the respective serotype. Viruses: APMV-1 (panel B), APMV-2 (panel C), APMV-3 (panel D), APMV-4 (panel E), APMV-5 (panel F), APMV-6 (panel G), APMV-7 (panel H), APMV-8 (panel I), APMV-9 (panel J), and mock-infected (panel A).

**Table 2:** Virus titers in the indicated tissue harvested from mice 3 dpi with APMV serotypes 1 to 9, expressed as mean fluorescent foci/gram of tissue.

APMV serotype	Lung	Nasal Turbinate	Brain
**1**	2×10^2^	3×10^1^	-
**2**	3×10^2^	6×10^1^	-
**3**	7×10^1^	2×10^1^	-
**4**	2×10^2^	1×10^2^	-
**5**	-	-	-
**6**	2×10^2^	3×10^2^	-
**7**	3×10^1^	1×10^1^	-
**8**	5×10^2^	2×10^2^	-
**9**	9×10^2^	8×10^2^	-

All the values are the mean of 3 mice per group.

*Titers were determined by serial dilution of clarified tissue homogenates from the experiment in Table 1 onto DF1 cells, which were overlaid with methylcellulose and immunostained 4 days later with N protein-specific antisera to detect viral foci.

-  = no virus was isolated.

### Immunonohistochemistry

The remaining half of each of the tissue samples isolated on 3 dpi and 14 dpi from the mice infected with the APMV serotypes was fixed and embedded in paraffin, and tissue sections were prepared. The tissue sections representing all of the collected tissue samples from the virus-infected and mock-infected animals from 3 dpi and 14 dpi were deparaffinized and immunostained using polyclonal antiserum specific to the N protein of the corresponding APMV serotype. Large amounts of APMV-specific N antigen was detected at 3 dpi by immunofluorescence staining of lungs and nasal turbinate tissue samples of mice infected with all the serotypes of APMV except serotype 5, which was negative (Fig. 3a and 3b). In the lungs of mice infected with each of the APMV serotypes except serotype 5, the viral antigen was localized mainly on the respiratory epithelium lining small and medium bronchi. In nasal turbinates of mice infected with each of the APMV serotypes except serotype 5, the virus specific immunoflourescence was observed on nasal epithelium lining the turbinate bone. No viral N antigen was detected in tissue samples from brain, spleen, kidney and small intestine of mice 3 dpi or 14 dpi with any the APMV serotypes, or from the lungs and nasal turbinates 14 dpi.

RETRACTED

**Figure 3:** Immunohistochemistry of sections of lungs (3a) and nasal turbinates (3b) harvested from mice 3 dpi with each of the 9 APMV serotypes. Mice were mock-infected (panel A) or infected with APMV-1 (panel B), APMV-2 (panel C), APMV-3 (panel D), APMV-4 (panel E), APMV-5 (panel F), APMV-6 (panel G), APMV-7 (panel H), APMV-8 (panel I), and APMV-9 (panel J). Immunofluoresence was performed with polyclonal antiserum specific to the respective serotype N protein (magnification, ×400). In sections of the lungs from mice infected with different APMVs, immunofluorescence was evident around the bronchial epithelium (Fig. 3a). In sections of the nasal turbinates from mice infected with different APMVs, immunofluorescence was evident around the bronchial epithelium, at the apical surface of the ciliated epithelial cells and in the cytoplasm (Fig. 3b). Bronchioles are shown by arrow.

### Histopathology

Tissue sections also were stained with hematoxylin and eosin and examined for histopathology. Lesions were observed in the lungs at 3 dpi in all the mice infected with each of the APMV serotypes except serotype 5, for which no histopathology was evident. Lesions were more severe in the alveoli and interstitial tissue, and were less severe in the airways. Severe multifocal to coalescing acute necrotizing bronchointerstitial pneumonia was noticed in lung tissues infected with APMV-1 and APMV-2, while mild to subacute bronchointerstitial pneumonia was observed in the other APMVs infected mice (Fig. 4). There was involvement of bronchiolar epithelium in some of the tissue samples. In some of the lung samples, alveolar hemorrhage and fibrin, which may be necrotizing, was observed. In addition, syncytia involving type II pneumocytes was evident for each of the APMVs except for APMV-4, APMV-5, and APMV-8 (Fig. 4 marked arrow). Microscopic lesions were not found in the lungs of any mouse at 14 dpi. In addition, lesions were not found in any other tissues on either day.

RETRACTED

**Figure 4:** Histopathology in sections of lungs harvested from mice 3 dpi with each of the APMV serotypes. Mice were mock-infected (panel A) or infected with APMV-1 (panel B), APMV-2 (panel C), APMV-3 (panel D), APMV-4 (panel E), APMV-5 (panel F), APMV-6 (panel G), APMV-7 (panel H), APMV-8 (panel I), and APMV-9 9panel J). Sections were stained with hematoxylin and eosin (magnification, ×400). In mock-infected mice, the bronchiole is lined by a single layer of epithelial cells, alveoli are filled with air (although partially collapsed) and lined by flattened type I pneumocytes and there is mild acute alveolar hemorrhage likely secondary to CO2 euthanasia. APMV-5 infected mice had no detectable lesions and were indistinguishable from mock-infected mice. In APMV-1 and -2 infected mice, severe subacute diffuse necrotizing bronchointerstitial pneumonia was observed (panels B and C). Further, alveolar spaces and septae are filled with hemorrhage, fibrin, edema, and mixed inflammatory cells (neutrophils, macrophages, lymphocytes, plasma cells), as well as necrotic cellular debris (panels B and C). In APMV-1 infected mice, alveolar spaces/interstitium are more severely affected than are the airways (panel B). Further, bronchiolar epithelial cells are hypertrophied with karyomegally and occasional individual cell necrosis/apoptosis was also observed (panel B). In APMV-7 and -9 infected mice, there is type II pneumocyte hypertrophy as well as endothelial cell hypertrophy (black arrows in panels H and J). In APMV-8 infected mice, there are neutrophils in expanded alveolar septae (black arrow in panel I). However, mild bronchointerstitial pneumonia was observed in mice infected with some APMVs with different degrees of bronchiole damage (panels D, E and G to J).

### Seroconversion

The sera of the mice infected with the different serotypes of APMV were collected at 14 dpi. Sera from mice infected with each of the APMV serotypes except serotype 5 were analyzed for virus-specific antibodies by a modified HI assay using chicken erythrocytes. The HI titers of the pre-infection and control mice were 2 or less. An HI titer of greater than 8 was considered positive. Every infected mouse seroconverted, indicating that viral replication had occurred (Table 3). The mean serum HI titers of mice infected with APMV serotypes 1, 2, 3, 4, 6, 7, 8 and 9 were 1∶64, 1∶64, 1∶64, 1∶16, 1∶16, 1∶64, 1∶64, 1∶64, respectively. In the case of APMV-5, which does not hemagglutinate, antibody titers were measured by a plaque reduction assay. However, none of the mice infected with APMV-5 developed detectable neutralizing serum antibodies.

RETRACTED

**Table 3:** Serum antibody responses against APMV serotypes 1–9 in infected mice^a^.

APMV serotype	HI antibody titer^b^
**1**	1∶64
**2**	1∶64
**3**	1∶64
**4**	1∶16
**5**	-
**6**	1∶16
**7**	1∶64
**8**	1∶64
**9**	1∶64

All the values are averages from three independent experiments.

a Mice in groups of 3 were inoculated as in Table 1. Serum samples were collected before inoculation and 14 dpi.

b The hemagglutination inhibition (HI) titer is expressed as the reciprocal of the highest serum dilution causing complete inhibition of four HA units of NDV.

-  = not detected.

## Discussion

APMVs are frequently isolated from wide variety of avian species around the world and have been grouped into nine serotypes based on antigenic relatedness involving the HN protein. Among the nine serotypes, APMV-1 (NDV) is the most studied member due to its importance as a major pathogen of poultry. APMV serotypes 2 to 9 are frequently isolated from both domestic and wild birds, but have been largely uncharacterized until recently. APMV-1 has been shown to infect not only avian species but also non-avian species, although its replication is restricted in non-avian hosts. APMV-1 is being developed as promising viral vaccine vector for delivery of a number of foreign antigens of animal and human pathogens. Further, APMV-1 has been developed as safe and effective oncolytic agent both in mouse models and also in human clinical trials [51]–[53], [57]–[59]. Therefore, it is of interest to also evaluate APMV serotypes 2 to 9 as potential vaccine vectors and oncolytic agents. However, the ability of APMV serotypes 2 to 9 to replicate in mammalian hosts was unknown.

The goal of this study was to evaluate intranasal infection by representative APMVs in mice to assess pathogenesis in a non-avian host and to identify a small laboratory animal model for further studies. Mice were evaluated for permissiveness to infection by APMV serotypes 1 to 9, clinical disease, magnitude and location of replication in the respiratory tract, dissemination to other tissues, disease, histopathology, and induction of antibodies. Inbred mice have been commonly used to study replication and pathogenesis of various viruses, to screen attenuation phenotypes of live virus vaccines, and to evaluate immune responses and protective efficacy elicited by virus vaccine candidates. This animal model is desirable for a number of reasons (i) Inbred mice represent a genetically homogenous model for which many reagents are available (ii) The degree of replication in the respiratory tract and other organs is readily measured (iii) Pathogenesis is readily monitored (iv) Innate, cellular, humoral and mucosal immune responses can be readily measured and (v) The mouse has the same body temperature as humans, and is a convenient mammalian host.

RETRACTED

In this study, we have evaluated the replication and pathogenicity of APMV serotypes 2 to 9 in mice by a natural (intranasal) route of infection. Mice infected with different serotypes of APMV showed relatively mild or no clinical signs. Mice infected with APMV serotypes 1, 2, 6, 7 and 9 exhibited loss of weight that was more marked with serotypes 1 and 2. However, these mice recovered fully by 7^th^ day of infection and showed no further clinical signs. The order of severity of clinical disease and weight loss was: 1, 2>6, 9>7. The other serotypes did not induce clinical disease. Mice infected with any of the APMV serotypes exhibited no gross pathological lesions in any of the organs.

Each of the APMV serotypes replicated to low-to-moderate titers in the lungs and nasal turbinates on 3 dpi except for serotype 5, for which infectious virus could not be recovered from any tissue at any time point. In the case of APMV serotypes 4 and 9, the brain tissue samples from two of the three infected mice in each group were positive for infectious virus 3 dpi when assayed in embryonated eggs, but were negative for virus recovery in cell culture. This suggests that the viral titers in the brain samples were very low. Infectious virus was not detected in any other tissue samples for any serotype. These findings indicate that replication by the APMV serotypes is largely restricted to the upper and lower respiratory tracts. In our study virus could not be detected in spleen in contrast to previous findings [60]. These discrepancies could be due to the differences in route of inoculation in two studies. Consistent with this, mild histopathological lesions were observed 3 dpi in the respiratory tract for all of the serotypes except APMV-5, which was negative. Lesions were not observed in any other tissues. Also, immunohistochemical staining detected viral N antigen in the lungs and nasal turbinates 3 dpi, but not in any other tissue. An interesting finding was the presence of large amounts of viral antigens at the epithelial cell linings, suggesting that these viruses have tropism towards the superficial layer of epithelial cells. On 14 dpi, virus was not detected in any of the tissues for any of the APMV serotypes, either by virus isolation or immunostaining. In addition, no histopathologic lesions remained. Thus, the infections had completely resolved by 14 dpi.

RETRACTED

The different APMV serotypes induced a spectrum of disease severity. At one extreme, mice infected with serotypes 1 and 2 exhibited ruffled fur, huddling, decreased physical activity, and substantial weight loss. At the other extreme, serotypes 3, 4, 5, and 8 did not exhibit any disease signs apart from marginal weight loss in some instances. Serotypes 6, 7, and 9 were intermediate in disease signs. The clinical disease that was observed was short-lived. Increased disease was not reflected by substantial increases in the titer of infectious virus recovered from the lungs and nasal turbinates. For example, APMV-1 and -2 induced the most clinical disease, but the viral titers observed with APMV-1 and -2 were similar to those with APMV-4, -6, -8, and -9 for which disease was either less (APMV-6 and -9) or not apparent (APMV-4 and -8). Similarly, the amount of antigen observed in the epithelial linings of the lungs and nasal turbinates was extensive for all of the viruses except APMV-5, and thus usually was not accompanied by severe disease. These findings are favorable with regard to the possible use of these viruses as vaccine vectors, since extensive antigen expression with minimal disease and minimal-to-moderate virus replication are desired characteristics. Serological analysis demonstrated a humoral response in the mice inoculated with different serotypes of APMVs except serotype 5, a further indication that APMV-5 did not replicate significantly. These results show that, with the exception of serotype 5, the APMVs are capable of infecting mice by the intranasal route with extensive antigen expression and minimal disease.

Previously, pathogenicity of APMV-3 strain Netherlands in 9-day-old embryonated chicken eggs, 1-day and 2-week-old chickens and turkeys was examined [41]. The mean death time (MDT) in 9-day-old embryonated chicken eggs was 112 h and intracerebral pathogeneicity index (ICPI) in 1-day-old chicks was 0.39. It caused mild respiratory disease in 1-day-old chickens and turkeys after inoculation through oculonasal route. In 2-week-old chicken and turkeys, it did not cause any disease. All the birds were seroconverted and the virus was detected in brain, lungs, alimentary tract, spleen, trachea, pancreas and kidney. Subbiah *et al*. [40] studied pathogenicity of APMV-2 strain Yucaipa in 9-day-old embryonated chicken eggs, 1-day and 4-week-old chickens and turkeys. The MDT in 9-day-old embryonated chicken eggs was more than 168 h and ICPI in 1-day-old chicks was zero. After oculonasal inoculation, it did not cause any disease in 4-week-old chickens and turkeys, although all the birds were seroconverted. The virus was detected in respiratory and alimentary tracts. In another study, experimental infection of 1-day-old chicks with APMV serotypes 2, 4 and 6 resulted in viral infection and virus was recovered from infected birds' trachea, lungs, gut, and pancreas [61]. Similar to the findings in chickens, we were able to detect the virus in respiratory tract of mice but we were not able to isolate infectious virus or detect viral antigen for any of the APMV serotypes in the spleen, kidney and small intestines of the mice, suggesting that the tropism of these APMVs is more restricted in mice, presumably reflecting reduced replication and host-range restriction in this non-avian species. However, the observation that trace amounts of APMV-4 and -9 were detected in the brain will need to be further evaluated.

RETRACTED

Our results identified BALB/c mice as a small animal model that supported replication in the respiratory tract of all of the APMVs except for APMV-5, which failed to infect detectably. Except for APMV-5, each APMV induced a substantial humoral immune response. The replication of APMVs in mice produced a spectrum of mild, short-lived disease that was restricted to the respiratory tract. These results suggest that, like APMV-1, the other APMV serotypes are candidates for evaluation in non-human primates as potential vaccine vectors attenuated by host rang restriction. In conclusion, this study is the first comparative report on the replication and pathogenicity of prototype strains of all nine APMV serotypes in mice. Our results lay the foundation for a good laboratory animal model for testing the replication and pathogenicity of APMV strains.
